# Position of the Hyoid Bone in Anteroposterior Skeletal Patterns

This article has been retracted.

**DOI:** 10.1155/2021/7130457

**Published:** 2021-08-30

**Authors:** Rabia Bilal

**Affiliations:** Department of Orthodontics Faculty of Dentistry, Qassim University Kingdom of Saudi Arabia, Buraydah, Saudi Arabia

## Abstract

**Introduction:**

Hyoid bone plays a vital role in the craniofacial dynamics. From the maintenance of pharyngeal airway to phonation, deglutition, and mandibular movements, it has multifactorial roles to fulfill. The hyoid bone has a spatial relationship with cranial base, mandible, and cervical vertebrae. This study was performed to determine the position of the hyoid bone in different anteroposterior growth patterns.

**Materials and Methods:**

75 lateral cephalograms belonging to all three sagittal skeletal patterns were evaluated in the study. The angular and linear measurements using 10 variables were made to determine the relationship of the hyoid bone with different craniofacial structures. SPSS was used to calculate the descriptive statistics, mean, and standard deviation of all the linear and angular variables. The analysis of variance (ANOVA) and post hoc test were used to compare the means of linear and angular measurement and multiple comparisons, respectively, at *p* < 0.05 significance level.

**Results:**

There was no significant difference in the mean angular measurements (NSH and MPH) between the 3 groups (*p* > 0.05). Also, the multiple comparisons showed no significant difference between the linear measurements (H-FH, H-MP, H-H′, and H-N). However, there was a significant difference in three linear measurements: H-Rgn, RGN-C3, and C3-H. The values were more in class III subjects, compared to class I and class II.

**Conclusion:**

The linear millimetric distance between points H-RGN, RGN-C3, and C3-H which determine the relationship and spatial position of the hyoid bone with the mandible and third cervical vertebrae was statistically significant among groups. The values were more in class III subjects inferring the anterior position of the hyoid bone.

## 1. Introduction

The hyoid bone is a small horseshoe-shaped solitary bone located below the mandible anteriorly in the midline of the neck. It connects the head and neck. It has a body, two lesser horns, and two greater horns. The hyoid bone keeps the pharyngeal airway open during sleep, phonation, and deglutition. It helps during the movement of mandible and maintains the position of tongue. Moreover, due to its complex connection between the mandible and the cervical spine, it maintains the posture of the head [1]. Despite not having any bony connection, it joins with tongue, mandible, cranial base, thyroid cartilage, sternum, pharynx, and scapula through supra and infrahyoid muscles. Due to these connections, any change in the position of these structures might have an effect on the position of the hyoid bone [2]. There is wide ranging literature on the functional anatomy, morphological characteristics, and diagnostic significance of the hyoid bone. Also, the relationship and anatomic position of the hyoid bone with cervicofacial structures are critically investigated. This depicts the importance of hyoid in the clinical orthodontics and dentofacial orthopedics [3]. Studies have also shown that the change in the position of the hyoid bone is related to the changes in mandibular position during mandibular movements [4, 5]. The position of the hyoid bone was studied by Battagel et al., who concluded that the hyoid bone was positioned more posteriorly in class II subjects with narrow upper airways [6]. On the contrary, a more anteriorly positioned hyoid bone was seen in class III subjects when compared to class I [7]. Literature also supports more the posteriorly placed hyoid bone in class I horizontal patterns as compared to anteriorly placed in the class III pattern [8].

Studies performed on the relationship of the hyoid bone with base of the skull and mandible demonstrated that the position of the hyoid bone varied in relation to the anterior cranial base of the skull. The hyoid bone was placed backward in class II subjects, while it was forward placed in class III subjects [9]. Manual change in the position of the mandible has also shown change in the position of the hyoid bone. Surgical advancement of mandible resulted in anterior positioning of the hyoid bone and widening of the minimal pharyngeal airway space [10], whereas surgical mandibular setback was associated with posterior positioning of hyoid and reduction of the sagittal dimensions of the oropharyngeal airway space [11].

Lateral cephalogram was introduced by Broadbent in 1931 and holds the colossal value in diagnostic and therapeutic orthodontics [12, 13]. Lateral cephalogram is a common tool used to measure the relationship and position of the hyoid bone with different anatomical structures of the head and neck [14]. Grabber suggested anatomical landmarks on lateral cephalogram specific to the assessment of hyoid bone position. The linear measurements and angles formed by joining those landmarks can help determine the position of the hyoid bone in static and dynamic state; also, it helps establish the relationship of the hyoid bone with the surrounding soft and hard tissues of the face and neck [15].

This study was performed to determine the position of the hyoid bone with reference to cranial base, maxilla, and mandible in anteroposterior plane in different horizontal growth patterns. This will give an insight to the hyoid pattern in people of this region and will help in better understanding of postural dynamics in clinical orthodontics.

## 2. Materials and Methods

The study was approved by the Ethical Committee of College of Dentistry, Qassim University (EA/6000/2017). The retrospective data were collected from the lateral cephalograms of the patients who presented to OPD clinics for the purpose of consultation or treatment at College of Dentistry. All the 75 lateral cephalograms were taken in a standardized manner in natural head position with Soredex Cranex *D* panorex + ceph X-ray machine, Tuusula, Finland.

All the selected cephalograms met the inclusion criteria, i.e., normal vertical growth pattern, age between 14 and 24 years, and showing clear craniofacial landmarks. Those with obstructive sleep apnea had underwent or undergoing orthodontic/orthognathic surgical treatment, systemic disease, congenital abnormality, or history of orofacial trauma were excluded from the study. The lateral cephalograms were divided into three sagittal groups: class I, class II, and class III on the basis of SNA, SNB, and ANB values. The anatomical landmarks were identified by putting the cephalograms on the X-ray view box. Cephalograms were manually traced on the TruVision cephalometric acetate tracing sheet (0.003″ thick, 8′x 10″ size) by Ortho Technology, Tampa, Florida, USA, with lead pencil. Landmarks were identified, planes were drawn, and linear and angular measurements were measured by two different observers. Interobserver reliability was determined by using Cohen's Kappa coefficient. *K* = 0.88 (*K* < 1). The *K* value shows a good agreement between the observers in identification of landmarks and measurement of planes and angles.

Intraobserver reliability was measured by asking the same observer to trace randomly selected 10 cephalograms after an interval of one week from the first measurements, and intraclass correlation coefficient (ICC) between first and second measurements was calculated. The tracing and landmark identification showed consistency of 99%.

The angular measurements followed are shown in Figure 1.

The linear measurements followed are shown in Figure 2.

## 3. Data Analysis

The data were analyzed using Statistical Package for Social Sciences (SPSS) version 22.0 (IBM Corp., Armonk, N.Y., USA). Descriptive statistics were used to calculate the frequency and percentage of different anteroposterior skeletal classes of the sample (Figure 3).

Also, descriptive statistics were used to calculate mean and standard deviation of all the linear and angular variables (Table 1).

The analysis of variance (ANOVA) and post hoc Tuckey test were used to compare the means of linear and angular measurement and multiple comparisons, respectively, at *p* < 0.05 significance level.

## 4. Results

There was no significant difference in the means of angular and linear measurements, except for three linear measurements, which are H-RGN, RGN-C3, and C3-H (Table 2).

The post hoc Tuckey intergroup comparison showed that the class III group had increased the mean length of H-RGn, RGn-C3, and C3-H as compared to class I and class II groups. The larger *F* values of these three linear readings also illustrate larger dispersion and variation in the class III group as compared to class I and class II, while there was no significant difference in class I and class II groups.

## 5. Discussion

The findings of this study do not suggest any statistically significant difference in the angular measurements of NSH and MPH angles (*p* > 0.05). The NSH is the angle formed between the cranial base and hyoid bone; hence, it depicts the position of the hyoid bone with reference to the cranial base. The insignificant difference in this study suggests that the position of the hyoid bone remains unchanged in different anteroposterior patterns. Also, the value of the MPH angle (the angle between the hyoid bone and mandibular plane) was insignificant, which shows there was no difference in backward and forward movement of the hyoid bone during the movement of lower jaw, although the bone is attached to the mandible through the suprahyoid muscles.

A study done by Amayeri showed different findings from our study. His study concluded that the angular measurements of NSH and MPH differed with different facial patterns. The hyoid bone moved backward in class II and moved forward in class III pattern [3]. Other studies also showed class II subjects having a posteriorly placed hyoid bone and class III subjects having the anteriorly placed hyoid bone [6, 7, 9]. These outcomes can be credited to the soft tissue pull between the hyoid and mandibular bones, responsible for the forward and backward movement of the hyoid bone during the jaw movements.

The insignificant difference between the values and sagittal class in our study suggests there was perhaps no significant change in the position of the hyoid bone during jaw movements. A study performed by Ingervall suggested that though some agreement exists on the backward movement of hyoid during cranial extension and forward movement during flexion, but mostly maintains its level, moving slightly backward during mandibular movement [16].

For the linear values, H-SN, H-FH, and H-MP perpendicular distance in mm was also not statistically significant (*p*=0.972, 0.844, and 0.449, respectively). These readings relate the hyoid bone with cranial base, Frankfurt horizontal, and mandibular plane, respectively. The insignificant values depict somewhat similar position of the hyoid bone in reference to these anatomical planes in all three anteroposterior classes. The linear millimetric distance of H-H′ and H-N, which relates the hyoid position with mandible and anterior cranial base, was also statistically insignificant.

Although in the study done by Amayeri et al. [3], the H-SN and H-FH were statistically significant, but the linear measurements in relation to the anterior cranial base in the anteroposterior direction (H-N perpendicular) was statistically insignificant among the study and control groups as exhibited in our study. This was in disagreement with a study conducted by Adamidis and Spyropoulos [7] who reported that the distance between the hyoid bone and the nasion was smaller in class III patients.

The linear millimetric distance between points H-RGn, RGn-C3, and C3-H determines the relationship and spatial position of the hyoid bone with the mandible and 3^rd^ cervical vertebrae. These measurements correlate the hyoid bone with mandible, mandible with C3, and C3 with the hyoid bone. This is integral in defining the position of the hyoid bone with lower jaw movements, postural activity of tongue, and width of upper airway. In our study, the distance was significantly larger in class III subjects (42.75 mm, 79.00 mm, and 38.75 mm) (*p*=0.000) as compared to class I and class II subjects, in which the distances were almost same. Same results were found in a study done by Amayeri et al. [3] in which the third vertebrae to the hyoid bone distance was statistically greater in class III as compared to class I and class II. The same result was found in a study performed by Ismail and Husamettin [17]. The authors concluded a reverse relationship between the ANB angle and H-C3 distance. Lesser angle was associated with larger distance. The study by Saleh and Nadeem [18] concluded that in subjects with raised ANB angle, the hyoid bone moved in a more posterior position. This illustrates that the smaller hyoid bone to third vertebrae distance will be seen in the class II sagittal pattern as compared to the class III pattern in which the distance will be increased. A study done by Mortazavi et al. [19] showed the similar results. They established that the anteriorly positioned hyoid bone makes the lower section of the upper airway wider.

An interesting study was performed on the skeletal class II growing subjects who were treated with an activator. This functional growth therapy resulted in a significant displacement of the hyoid bone in anterior direction; also, the linear distance between hyoidale and the third cervical vertebrae (C3-H) was increased. The linear distance between the mandible from retrognathion and the third cervical vertebrae (RGn-C3) was also significantly increased [20–22].

All these outcomes are same as the findings of our study and also those found in literature, in which the linear measurements are lesser in class II and class I subjects as compared to class III. This perhaps explains short upper airway dimensions in class II and obstructive sleep apneic patients, where the mandible and hyoid bones are posteriorly placed, and subsequent distances between the hyoid bone, RGn, and C3 are reduced. The opposite holds true for class III subjects.

Most of the studies on the hyoid bone are done on Caucasian, Orientals, and South American population. There does not exists ample information on the position of the hyoid bone in Saudi population. This study gave an important insight on the hyoid bone in Saudi populace. More studies with larger samples are recommended for a more comprehensive information on the role of the hyoid bone in orthodontics and dentofacial orthopedics.

## 6. Conclusion

The findings of this study do not suggest any statistically significant difference in the angular measurements of NSH and MPH angles. The linear distances H-SN, H-FH, and H-MP are perpendicular, and also, H-H′ and H-N were statistically insignificant. However, the linear distance between points H-RGn, RGn-C3, and C3-H which determine the relationship and spatial position of the hyoid bone with the mandible and C3 was statistically significant in all groups. The values were more in class III subjects; this shows the anterior position of the hyoid bone in the class III pattern as compared to class I and class II. This is an important finding which should be borne in mind while performing the orthopedic and orthognathic treatment modalities on patients of this region, as the position of the hyoid bone plays an important role in postural dynamics in clinical orthodontics. Further studies with a larger sample size and more diverse inclusion of various regions across kingdom are recommended.

## Figures and Tables

**Figure 1:** The angular measurements used to determine the position of the hyoid bone.

**Figure 2:** The landmarks and linear measurements used in the study.

**Figure 3:** The frequency and percentage of different sagittal classes.

**Table 1:** Showing the means of angular and linear measurements.

Angular and linear measurements	Class I	Class II	Class III
	Mean	Mean	Mean
NSH (angle)	90.79°	89.99°	87.30°
MPH (angle)	18.68°	19.76°	14.55°
H_SN (linear distance)	78.44 mm	77.95 mm	79.10 mm
H_FH (linear distance)	62.99 mm	63.46 mm	61.08 mm
H_MP (linear distance)	11.72 mm	11.98 mm	8.73 mm
H_H (linear distance)	4.22 mm	4.10 mm	1.99 mm
H_N (linear distance)	48.33 mm	45.76 mm	48.30 mm
H_RGN (linear distance)	35.99 mm	37.02 mm	42.95 mm
RGN_C3 (linear distance)	69.88 mm	70.08 mm	79.09 mm
C3_H (linear distance)	34.98 mm	34.06 mm	38.81 mm

**Table 2:** The multiple comparisons by ANOVA and post hoc Tuckey test.

Angular and linear measurements	Sum of squares	df	Mean square	*F* statistic	Significance
NSH	45.9	2	22.9	0.127	0.984
MPH	83.3	2	41.6	0.701	0.505
H_SN	4.6	2	2.3	0.028	0.977
H_FH	17.5	2	8.7	0.170	0.848
H_MP	35.5	2	17.7	0.814	0.454
H_H′	20.4	2	10.2	0.628	0.541
H_N	64.8	2	32.4	0.249	0.783
H_RGN	167.1	2	83.6	240.4	0.000^*∗*^
RGN_C3	3111.2	2	155.6	123.5	0.000^*∗*^
C3_H	69.5	2	34.7	64.4	0.000^*∗*^

^∗^Statistically significant difference.

## Data Availability

The data used to support the findings of this study are available from the author upon request.
